# An Overview of Supervised Machine Learning Methods and Data Analysis for COVID-19 Detection

**DOI:** 10.1155/2021/4733167

**Published:** 2021-11-22

**Authors:** Aurelle Tchagna Kouanou, Thomas Mih Attia, Cyrille Feudjio, Anges Fleurio Djeumo, Adèle Ngo Mouelas, Mendel Patrice Nzogang, Christian Tchito Tchapga, Daniel Tchiotsop

**Affiliations:** ^1^Department of Computer Engineering, College of Technology, University of Buea, Buea, Cameroon; ^2^Department of Training, Research Development and Innovation, InchTech's Solutions, Yaoundé, Cameroon; ^3^Department of Electrical and Electronic Engineering, College of Technology, University of Buea, Buea, Cameroon; ^4^Ecole Nationale Supérieur Polytechnique, University of Yaounde 1, Yaoundé, Cameroon; ^5^Faculté de Médecine et des Sciences Biomédicales, University of Yaounde 1, Yaoundé, Cameroon; ^6^Unité de Recherche d'Automatique et d'informatique Appliquée (UR-AIA), IUT-FV de Bandjoun, Université de Dschang-Cameroun, BP 134, Bandjoun, Cameroon

## Abstract

**Methods:**

Our analysis and machine learning algorithm is based on most cited two clinical datasets from the literature: one from San Raffaele Hospital Milan Italia and the other from Hospital Israelita Albert Einstein São Paulo Brasilia. The datasets were processed to select the best features that most influence the target, and it turned out that almost all of them are blood parameters. EDA (Exploratory Data Analysis) methods were applied to the datasets, and a comparative study of supervised machine learning models was done, after which the support vector machine (SVM) was selected as the one with the best performance.

**Results:**

SVM being the best performant is used as our proposed supervised machine learning algorithm. An accuracy of 99.29%, sensitivity of 92.79%, and specificity of 100% were obtained with the dataset from Kaggle (https://www.kaggle.com/einsteindata4u/covid19) after applying optimization to SVM. The same procedure and work were performed with the dataset taken from San Raffaele Hospital (https://zenodo.org/record/3886927#.YIluB5AzbMV). Once more, the SVM presented the best performance among other machine learning algorithms, and 92.86%, 93.55%, and 90.91% for accuracy, sensitivity, and specificity, respectively, were obtained.

**Conclusion:**

The obtained results, when compared with others from the literature based on these same datasets, are superior, leading us to conclude that our proposed solution is reliable for the COVID-19 diagnosis.

## 1. Introduction

The novel coronavirus known as SARS-CoV-2 (Severe Acute Respiratory Syndrome), responsible for COVID-19 pandemic, belongs to the large family of coronaviruses that cause fever, cough, dyspnea, and muscle pain, while imaging frequently reveals bilateral pneumonia [1–3]. Although the WHO validated an anti-COVID-19 vaccine [4], it cannot help alone to reduce the spread of the virus. Usually, the standard diagnostic method used is real-time reverse transcription-polymerase chain reaction (RT-PCR), which can help detect viral nucleosides in samples obtained from oropharyngeal swabs, nasopharyngeal swabs, bronchoalveolar washes, or tracheal aspirates acid [5–7]. Due to the constraints imposed by the latter, several health centers are opting for immunological or antibodies tests as an alternative [8]. However, these tests do not detect the presence of the virus, but rather the presence of IgM (Immunoglobulin M) and IgG (Immunoglobulin G) antibodies, produced to fight the virus. It is almost impossible to detect these antibodies before fourteen days after infection, this can lead to false-negative results (false negatives) [9, 10]. Faced with these limitations, health specialists have seen fit to call on scientists to obtain faster, more efficient, accessible, and more pleasant technological solutions.

Many researches are focusing on artificial intelligence (AI) technologies, machine learning (ML), and deep learning (DL) to deal with COVID-19 [11–14]. For example, ML algorithms have been used to detect COVID-19 CT-scans images from the lung [15]. In [16, 17], authors have shown that chest CTs are highly sensitive to the diagnosis of COVID-19. Due to the radiation dose, the relatively small number of available equipment, and the associated operating costs, CT-scan imaging can hardly be used for screening tasks. Furthermore, this method has obvious abnormalities when the lungs are inflamed or have tissue lesions [18]. A similar article on chest X-rays, which is a less expensive and low-dose test, was recently published with encouraging statistical performance [19]. However, it has been found that almost 60% of the chest X-rays taken by patients diagnosed with symptomatic COVID-19 are normal, and the system based on this examination needs to be thoroughly verified in the actual environment [20, 21]. Despite these encouraging results, they still attract some attention. Most of the other works have not yet been peer-reviewed: a recent important survey report stated that all surveyed studies may have a high risk of bias and overfitting and almost fail to comply with reporting and reproduction standards [22, 23]. Because of the aforementioned limitations of CT scan, RT-PCR, and immunological or antibodies test methods, there is an urgent need to seek for a more efficient and faster method for the detection of COVID-19.

In this paper, we propose an alternative method of testing based on data analysis (DA) and ML algorithms that are rapid, accessible, simple to use, and of low cost and have good accuracy. Our solution is designed to quickly and reliably predict whether or not an individual is infected by SARS-CoV-2 based on clinical data from individuals who have performed PCR tests. To perform this work, the datasets are transformed into a suitable format by using DA methods and then using ML; the best-correlated features with the target are retained. Secondly, a suitable model by which the data will be trained is determined, and finally, the model is optimized so to achieve the best performance.

The rest of our work is organized as follows.  Section 2 presents the state of the art of the related works carried out.  Section 3 deals with the DA and ML methods used, mainly the different methods used to carry out our work.  Section 4 presents the obtained results and discussions and comparisons with related works. This work ends in Section 5 with the conclusion and suggested future work.

## 2. Related Works

Several works based on AI, along with ML and DL, have been carried out over the last two years in the context of diagnosis and detection of COVID-19 infections. In this section, we will present some related works, including the models and methods that authors have used, and their results show the difference between the respective works and our proposed work.

Brinati et al. [23] proposed a feasibility study using ML algorithms detection of COVID-19 infection from blood exams with ML. The authors developed two ML classifiers based on hematochemical values (usual blood exams) from two hundred and seventy-nine (279) types of data from [24]. They proposed ML classifiers discriminated between patients who are either negative or positive to the SARS-CoV-2: their accuracy spectrum between 82% and 86% and sensitivity between 92% and 95% relative to the gold standard. In 2020, Soares et al. [25] proposed a novel specific artificial intelligence-based method to identify COVID-19 cases using simple blood exams. They developed a machine learning classifier that takes widely available simple blood exams as input and classifies samples as likely to be positive (having SARS-CoV-2) or negative (not having SARS-CoV-2). Based on this initial classification, positive cases can be referred for further highly sensitive testing (e.g., CT scan or specific antibodies). They used publicly available data from the Albert Einstein Hospital in Brazil from 5,644 patients. Focusing on simple blood exam figures as main predictors, 599 subjects that had the fewest missing values for 16 common exams were selected. From these 599 patients, 81 tested positive for SARS-CoV-2 (determined by RT-PCR). Based on the reduced dataset, they built an artificial intelligence classification framework, ER-CoV, aiming at determining if suspect patients arriving in ER were likely to be negative for SARS-CoV-2, that is, to predict if that suspect patient is negative for COVID-19. The primary goal of this investigation is to develop a classifier with high specificity and high negative predictive values, with reasonable sensitivity. Banerjee et al. [26] proposed the use of artificial intelligence (AI) along with ML to predict COVID-19 from blood samples. They collected SARS-CoV-2 rt-PCR samples with anonymized full blood counts results from Hospital Israelita Albert Einstein, in São Paulo, Brazil. They found that, with full blood counts, shallow learning, random forest, and artificial neural network model predict SARS-CoV-2 patients with high accuracy between populations on regular wards (AUC = 94–95%) and those not admitted in the community or to the hospital or AUC = 80–86% [26]. In 2020, Moraes Batista et al. [27] investigated ML to diagnose and predict COVID-19 for emergency patients. The authors based their investigation on the same dataset of authors from [26] and on five ML algorithms (neural networks, gradient boosting trees, random forests, support vector machines, and logistic regression) and trained their model. Their best predictive model was obtained by the SVM algorithm (AUC: 0.85; sensitivity: 0.68; specificity: 0.85; Brier Score: 0.16) that is not very reliable.

Freitas Barbosa et al. [28] based also on blood tests to develop an intelligent system to diagnose COVID-19 tested several ML methods to achieve high classification performance: 95.159% ± 0.693 of overall accuracy, sensitivity of 0.968 ± 0.007, kappa index of 0.903 ± 0.014, specificity of 0.936 ± 0.011, and precision of 0.938 ± 0.010. Their best results were achieved using Bayes Network and low computational cost classifiers. Soltan et al. [29] applied extreme gradient boosted trees, random forests, and multivariate logistic regression to distinguish admissions due to COVID-19 and emergency department presentations from prepandemic controls. They investigated the stepwise addition of clinical feature sets and assessed performance using stratified 10-fold cross-validation. Models were calibrated during training to achieve sensitivities of 70, 80, and 90% for identifying patients with COVID-19. They generated test sets with varying prevalence rates of COVID-19 and assessed predictive values to simulate real-world performance at different stages of the epidemic. Kukar et al. [30] based on ML proposed a COVID-19 diagnosis by routine blood tests. They constructed an ML predictive model for COVID-19 diagnosis. The model was based and cross-validated on the routine blood tests of 5,333 patients with various bacterial and viral infections. They selected an operational ROC point at a specificity of 97.9% and sensitivity of 81.9%, and the AUC was 0.97. According to the feature importance scoring of the XGBoost algorithm, the authors presented the five most useful routine blood parameters for COVID-19: prothrombin, albumin, eosinophil count, INR, and MCHC.

In 2021, AlJame et al. [31] used routine blood tests and proposed an ensemble learning model for COVID-19 diagnosis. For data preparation, they exploited a K-Nearest Neighbors algorithm to deal with null values in the dataset and an isolation forest method to remove outlier data. The proposed model was trained and evaluated by using publicly available data from [32]. The ensemble model achieved outstanding performance with an overall accuracy of 99.88%. Alves et al. [33] proposed also an ML model to diagnose COVID-19 from blood tests. The authors tested different ML models in a public dataset always from [32]. After performing data wrangling, this dataset had 608 patients, of which 84 were positive for COVID-19 confirmed by RT-PCR. By using random forest (RF) as their best ML algorithm, they achieved a good result (accuracy 0.88, F1–score 0.76, sensitivity 0.66, specificity 0.91, and AUROC 0.86).

Li et al. [34] also investigated COVID-19 detection by using ML algorithms. They found several novel associations between clinical variables, including the association between men and higher levels of serum lymphocytes and neutrophils. They found that COVID-19 patients can be divided into subtypes based on the serum levels of immune cells, gender, and reported symptoms. Finally, they trained an XGBoost model that can distinguish COVID-19 patients from influenza patients with a sensitivity of 92.5% and a specificity of 97.9%. Many other works have been performed in ML and blood samples in order to detect COVID-19 [35–43]. Others [44–47] explain how we can apply ML and DA on blood samples.  Table 1 summarizes the performance and description of related works. It can be observed in this table that the datasets from [24, 32] are widely used in the literature; that is why we used these datasets in our study and why at the end we compare our results with other results from the literature studies that have used the same datasets.

Despite these encouraging results as observed in Table 1, there are some concerns on the reliability, efficiency, and accuracy of their results. Also, we notice that the ML models are different for all the authors, and a model cannot give a good performance to each data set. Moreover, none of the authors in the literature has used DA and ML along with SVM to reach a very good performance in terms of rapidity, accuracy, specificity, and sensitivity. In this paper, therefore, we propose a method of analysis based on DA and ML techniques to analyze and select the best features for our ML algorithm. We optimize the SVM algorithm to finally have a performance superior to all algorithms found in the literature using the same datasets.

## 3. Proposed Approach

In this section, we give a detailed presentation of the different steps and methods used to carry out our work. Then, we first present our proposed pipeline. Afterward, we present the methods used for data analysis and exploration, data preprocessing, and data modeling. Finally, the optimization of the chosen model is presented.

Figure 1 presents our proposed pipeline that contains steps involved in the realization of our solution.

### 3.1. Exploratory Data Analysis

#### 3.1.1. Data Description

Our analysis is based on the dataset from [32]. This dataset contains the data of 5644 patients who performed a PCR test. These data are the parameter values obtained after analysis of the patients' blood and tests for the presence of already known viruses. In total, we have 111 features, and the target is represented by the variable *SARS-CoV-2 exam result*, which contains the results of the COVID-19 test carried out on the different patients.

#### 3.1.2. Deep Analysis of the Data Set

We divided the features into two different categories: blood (representing the features that were obtained from a blood test) and viral (representing the features that were obtained from a virological test). To visualize our data set before performing analysis, we have plotted some graphs.  Figure 2 shows the distribution of four features in our dataset while Figure 3 represents the relationship between the target and four features (viral) also and Figure 4 shows the relationship between blood feature and target.

*(1) Distribution of Continue Variables*. Blood type variables: blood.

 The majority of float variables follow the reduced Gaussian distribution. It is possible they have been standardized before in order to facilitate predictions.

*(2) Features-Target Relations*. Viral-target relation:

Looking at these figures, there are very few cases of double disease (people infected with both the SARS-CoV-2 virus and other viruses). On the other hand, the number of double negative cases is high (cases where patients are neither infected with SARS-CoV-2 nor other types of viruses). This suggests that if we do not have any infection of these other viruses, then it is highly likely that we are not infected with the SARS-CoV-2 virus.

*(3) Blood-Target Relation*.

From the previous figures, we can make the difference between the distribution of the positive and negative cases depending on each feature. The represented features have a great impact on the target. This proves that blood features have a great influence on the prediction of SARS-CoV-2 infection [35–37].

### 3.2. Data Preprocessing

The preprocessing starts by cleaning the dataset to select the best features.  Figure 5 shows the pipeline of the preprocessing step.

- **Cleaning**: It consists of deleting variables that have at least 90% of missing values. This new data set has the dimension (5644.32) and contains 10% positive cases and 90% negative cases.
- **Encoding:** Here, the target is to associate each qualitative value to a numerical value.
- **Imputation**: It consists of deleting or replacing missing values with other values in order to facilitate future operations.
- **Standardization**: It consists of putting all the variables (features and target) under the same scale by making them follow the same law of probability.
- **Features selection**: It consists of determining, using statistical methods, the ten feature variables that have the best impact on the target (SARS-CoV-2 exam result): we use the ANOVA (Analysis of Variance) statistical test to give the scores of the relationships between each feature and the target [38–40].

(1) $$\begin{array}{c} S_{1}=\overset{n_{\text{groupes}}}{\underset{1}{\sum }}n_{obs}\left[{\left(\bar{x}-µ\right)}^{2}+{\left(\bar{y}-µ\right)}^{2}\right],\\ S_{2}=\overset{n_{obs}-1}{\underset{i=0}{\sum }}{\left(x_{i}-\bar{x}\right)}^{2}+{\left(y_{i}-\bar{y}\right)}^{2},\\ D_{1}=\;n_{\text{groupes}}-1,\\ V_{2}=\frac{S_{1}}{D_{1}},\\ D_{2}=n_{obs}-n_{\text{groupes}},\\ V_{2}=\frac{S_{2}}{D_{2}},\\ F=\frac{V_{1}}{V_{2}}, \end{array}$$

where *n*_groupes_ is the number of groups. In our case, it is 2, because we calculate the ANOVA F score between each feature and the target, therefore, between two elements. *n*_*obs*_ is the number of observations in each feature. In our case, it is identical to the number of observations in the target; $\bar{x},\bar{y}$ are the average of the observations in any feature *x* and in the target *y*, respectively; *µ* is the average of the observations of the set made up of the different observations of *x* and *y*; *x*_*i*_, *y*_*i*_ are the observation of any feature *x* and target *y*.

Figure 6 shows the importance of each feature by using the ANOVA test.

We have selected the ten first ones to train and evaluate models.

The data set treatment phase has been achieved; it is now left to submit this to the different machine learning models to obtain the predictions.

### 3.3. Data Modeling

Data modeling can be seen as the process of creating an ML model for our dataset. Here, modeling starts with the choice of the training algorithm, followed by the metric evaluation. Based on the metric evaluation, we can choose the best algorithm for its optimization.  Figure 7 shows the pipeline of the modeling step.

#### 3.3.1. Models

We choose five high-performance classification models for small data sets (less than 100,000 lines), in particular, the KNeighbors classifier, bagging classifier, boosting classifier, SVM, and random forest classifier.

#### 3.3.2. Training

80% of the data set will be used as a train set or training data.

#### 3.3.3. Evaluation

20% will constitute the test set or data for evaluation or validation. The evaluation criteria are accuracy, precision, and recall.

(2) $$\begin{array}{c} \text{accuracy}\left(y,y_{\text{pred}}\right)=\frac{1}{n_{\text{samples}}}\overset{n_{\text{samples}}-1}{\underset{i=0}{\sum }}1\left(y_{{\text{pred}}_{i}}=y_{i}\right),\\ \text{recall}=\frac{\sum \text{True positive}}{\sum \text{True positive}+\sum \text{false negative}},\\ \text{specificity}=\frac{\sum \text{True negative}}{\sum \text{True negative}+\sum \text{False positive}}, \end{array}$$

where *n*_samples_ is the number of samples. *y*_pred_*i*__ is the predicted value of the *i*-th sample. *y*_*i*_ is the corresponding true value.

At the end of these 3 stages, the best model is selected, i.e., the one with the best performance.

### 3.4. Optimization of the Best Model

Optimization aims at improving the performance of the best model using the GridsearchCV technique.  Figure 8 shows the pipeline of optimization.

After giving a range of values to the hyperparameters of our best model, we train it with the GridSearchCV method. GridSearchCV is a technique that allows you to search within a range of hyperparameter values of a model, the optimal combination of values, allowing you to obtain better performance. The optimization is done by the *cross-validation* technique [41, 42]. After training, the hyperparameters have their optimum values. We then have an optimal best model, and we apply the evaluation criteria to obtain its performance.

### 3.5. Classification with SVM (Our Best COVID-19 ML Algorithm)

From [48, 49], given a training dataset *S*={(*x*_1_, *y*_1_),…, (*x*_*p*_, *y*_*p*_)} of data point *x*_*j*_ (with *X*⊆*ℝ*^*n*^) with matching labels *y*_*j*_ (with *Y*={−1, +1}), the task of COVID-19 classification here is to learn a function *h* : *X*⟶*Y* that properly classifies new examples (*x*, *y*) (*h* (*x*) = *y*).

A good classifier/model should guarantee the top possible generalization performance (minimum error on unseen examples) [48–50]. In SVM, the hyperplane found in the characteristic space matches the nonlinear decision borderline in the input space.

Let us consider in this case *ϕ* : *I*⊆*ℝ*^*n*^⟶*F*⊆*ℝ*^*n*^ a mapping from the input space *I* to the characteristic space *F*. In the learning step, the algorithm will find the hyperplane defined by the equation 〈*w*, *ϕ*(*x*_*j*_)〉=*b* such that the margin

(3) $$\begin{array}{c} y=\min_{1\leq j\leq p}y_{j}\left(\langle w,\phi \left(x_{j}\right)-b\rangle \right)=\min_{1\leq j\leq p}y_{j}h\left(x_{i}\right) \end{array}$$

is maximized, where 〈, 〉 denotes the inner product, *w* is a *p*-dimensional vector of weights, and *b* is a threshold. The quantity (〈*w*, *ϕ*(*x*_*j*_) − *b*〉)/‖*w*‖ represents the distance of the sample *x*_*j*_ from the hyperplane. It gives a positive or negative value for corrected and uncorrected classification, respectively, when multiplied by the label *y*_*j*_. A new data point *x* a label will be assigned to evaluate the decision function given by

(4) $$\begin{array}{c} h\left(x\right)=\text{sign}\left(\langle w,\phi \left(x_{j}\right)-b\rangle \right). \end{array}$$

In this paper, we work on the blood sample dataset and how we can base our investigation on this dataset to build a model able to detect if someone has COVID-19 or not. For that, we need to maximize the margin.

For linearly separable classes, there exists a hyperplane (*w*, *b*) given by

(5) $$\begin{array}{c} y_{j}\left(\langle w,\phi \left(x_{j}\right)-b\rangle \right)\geq \gamma ,\;j=1,\ldots ,p. \end{array}$$

By taking ‖*w*‖^2^=1, choosing a hyperplane to maximize the margin is equal to the following optimization problem:

(6) $$\begin{array}{c} y_{j}\left(\langle w,\phi \left(x_{j}\right)-b\rangle \right)\geq \gamma ,\;j=1,\ldots ,p. \end{array}$$

Problem (6) can be rewritten by using the Lagrange multipliers *α*_*j*_, *j*=1,…, *p* in the dual form given by

(7) $$\begin{array}{c} \max_{\alpha }\overset{p}{\underset{j=1}{\sum }}\alpha_{j}-\overset{p}{\underset{j=1}{\sum }}\overset{p}{\underset{k=1}{\sum }}\alpha_{j}\alpha_{k}y_{j}y_{k}\langle \phi \left(x_{j}\right),\phi \left(x_{k}\right)\rangle ,\\ \overset{p}{\underset{j=1}{\sum }}\alpha_{j}y_{j}=0,\;\alpha_{i}\geq 0. \end{array}$$

Problem (7) shows how to reduce a quadratic optimization task. However, the Karush–Kuhn–Tucker (KKT) conditions will be satisfied by the solutions *α*^*∗*^ ensuring that only a subset of training examples is associated with nonzero *α*_*j*_,  *j*=1,…, *p*. This property is crucial in our blood sample classification for COVID-19 detection and is called *sparseness of SVM.*

In the solution *α*^*∗*^, often only a subset of training examples is associated with nonzero *α*_*j*_,  *j*=1,…, *p*. These are called support vectors and correspond to the points that lie closest to the separating hyperplane (Fig.). For the maximal margin hyperplane, the weight vector *w*^*∗*^ is given by the linear function of the training points given by

(8) $$\begin{array}{c} w^{*}=\overset{p}{\underset{j=1}{\sum }}\alpha_{j}y_{j}\phi \left(x_{j}\right). \end{array}$$

Based on equation (8), equation (4) can be expressed in equation (9) as

(9) $$\begin{array}{c} h\left(x\right)=\text{sign}\left(\overset{p}{\underset{j=1}{\sum }}\alpha_{j}{}^{*}y_{j}\langle \phi \left(x_{j}\right),\phi \left(x\right)\rangle -b\right). \end{array}$$

For a support vector *x*_*j*_, it is (〈*w*^*∗*^, *ϕ*(*x*_*j*_)〉 − *b*)=*y*_*j*_ *j*=1,…, *p* from which the optimum bias *b*^*∗*^ can be computed.

To choose the best kernel function in SVM to deal with practical problems, we have the following [43]:

- Based on the prior knowledge of experts, we select the kernel functions
- The method of cross-validation is adopted; that is, when selecting the kernel function, different kernel functions should be tried, respectively, and the kernel function with the smallest error is the best kernel function

In this paper, we implement the SVM with RBF kernel in our algorithm.

## 4. Results

### 4.1. Modeling Results

After training our models, we get the learning curves of the different models as done in [43, 44].

These include the following:

- A training curve which gives the score after training (on the training sample) (Figure 9)
- A validation curve which gives the score after validation (on the validation sample) (Figure 9)

The first remark is that there is no convergence between the learning and validation curves. Random forest, bagging, and AdaBoost classifier are in overfitting [51]. The predictions are perfect on training (blue curve) but poor on validation (orange curve). To resolve this, we can cross-validate them on different splits. The curves of SVM seem to converge; this needs more training data.

In the next step, we observe the performance of each classifier after evaluation.

#### 4.1.1. Results after Evaluation on the Test Set

*(1) Performance Criteria of the Fives Models*. The performance criteria of the different models are obtained by computing the value of each metric.  Table 2 presents the values of metrics for each estimator.

After observing these values, we can say that the model with the best performance is SVM. Let us better appreciate this by observing the accuracy, precision, and recall curves in Figure 10.

We can notice that whatever the performance criteria, the SVM model has the highest score, in terms of accuracy, sensitivity, or specificity, which makes it the best model. All that remains now is to optimize it.

### 4.2. Optimization Results of the Best Model

#### 4.2.1. Training Results

After training the best model using the GridSearchCV method we obtained, we observe the learning curves presented in Figure 11.

We notice that there is no difference between this new model's learning curves and the former one. Perhaps, the hyperparameters of the former model are already the best. There is no need to modify it. This will be verified after observing the new confusion matrix.

#### 4.2.2. Results after Evaluation of the Optimized Best Model

In ML, the confusion matrix (also called the error matrix) is a specific table layout that can visualize the performance of the hypothetical algorithm we use, that is, the parameters of the SVM algorithm (negatively predicted number, positively predicted number). The confusion matrix of our optimized model is displayed in Table 3.

The model has very few false negatives (0.71%) and no false positives (0%); it does not make too much confusion between the two classes. This explains his high performance. Moreover, there is no difference between nonoptimized and optimized models: accuracy = 0.992, sensitivity = 0.927, and specificity = 1. So, our SVM model is very reliable and efficient.

### 4.3. Discussions

#### 4.3.1. Comparison with the Performance of Related Works

Figure 12 highlights the performance of our solution and the work of the authors cited in the literature review who worked on the same dataset [32] as ours.

As can be observed, the performance of our model is almost the highest in terms of accuracy and specificity. This performance may be due to the technique of choice of our final model, which started with the evaluation of several models, and then the choice of the best model. On the other hand, if we take a look at the other results, we will realize that there are solutions that perform better than ours mostly in terms of accuracy and sensitivity, even though we did not work on the same data set. This is the case of the solution resulting from the work [31], which reached 99.88%, 98.72%, and 99.99%, respectively, in terms of accuracy, sensitivity, and specificity.

We can confirm that our model is very efficient but is not perfect. In particular, this perfection is not achieved especially at the sensitivity level, which also affects the accuracy and prevents it from reaching value 1. Indeed, the achievement of this level of sensitivity (below 95%) can be explained by the low number of patients testing positive (only 10%) in our data set. This implies that the model was not trained on a large sample of positive cases, which affects the predictions of positive cases and lowers their performance. Sensitivity, being the ability to find all positive results, is therefore deteriorated.

In order to see if our DA and SVM method is good, we have carried out the same study using another dataset taken from [24] that contains one more parameter CRP (C-reactive protein). The SVM model once more has been the best model in terms of accuracy, sensitivity, and specificity. In Figure 13, we easily appreciate the best model depending on each metric. In this figure, we perform the representation of accuracy, specificity, and sensitivity.

According to Figures 13(a)–13(c), the SVM model has the best performance compared to the others. It achieved 92.86 of accuracy, 93.55 of sensitivity, and 90.91 of specificity. We then compared our result with the result from [23], who worked on the same dataset, and Figure 14 presents the difference between our models.

Although the sensitivity of [23] is higher than ours, the latter achieves 82–86% accuracy, which is under the accuracy of our model. This means that our model makes less errors in its prediction than the author's model from [23].

Regarding the discussions, we confirm that the results of the SVM model are good, either in the first or in the second dataset. Hence, it is important for us to find ways and means to improve the performance of our solution especially the sensitivity.

In a nutshell, we have presented the major results of the proposed solution, obtained during the modeling and evaluation stages. Based on performance (accuracy, precision, and sensitivity), we selected the best model among the five initially considered, and then, we improved its performance to be the best possible. We obtained very high performance on the test set: 99.29%, 92.79%, and 100% for accuracy, sensitivity, and specificity, respectively, concerning the first dataset (data set from [32]) and 92.86%, 93.55%, and 90.91% for accuracy, sensitivity, and specificity, respectively, concerning the second dataset (data set from [24]). By using our model, we can now perform a cheap COVID-19 test within less time. Furthermore, we can try to improve our model with some big data analysis techniques and tools used in biomedical engineering and presented in [52–54].

## 5. Conclusion

This study focused on the implementation of a solution to predict whether or not an individual is infected with SARS-CoV-2 quickly and reliably, based on DA and ML model as well as clinical data from patients who have carried out PCR tests. With a view to achieving these ends, we, first of all, presented some diagnostic works on COVID-19 already carried out. Then, we amply presented the approach used to achieve this solution. It began with an analysis and exploration of the data in order to understand our data set in depth. After understanding our data, we processed it in order to put it in a suitable format for machine learning. This processing consisted of encoding, imputation, standardization, and selection of the 10 best variables. The next step was modeling, in which we presented the five models to be trained and evaluated according to well-defined evaluation criteria, with the aim of selecting the best model. Finally, the last step was optimization, in which we used the “GridSearchCV” method, an optimization technique to increase the performance of the selected model. In the last part of this work, we highlighted the results obtained after the modeling and optimization phases, as well as extensive discussions. After training and evaluation of the different models, we selected the “SVM” as the best model, and then, we optimized it. At the end of the optimization, we observed that the performance remained the same: an accuracy of 0.99, a recall of 0.93, and a perfect specificity of 1. We did the same work with another dataset taken from [24]. Once more, the SVM presented the best performance: 92.86%, 93.55%, and 90.91% for accuracy, sensitivity, and specificity, respectively. At this point, we can easily say that blood parameters are a very good option to predict SARS-CoV-2 infection at low cost and rapidly. Our solution has several advantages, namely:

- Absence of costs related to the manufacture and transport of the tests
- Low dependence on qualified professionals for its use
- More pleasant for patients compared to the PCR test
- Accessibility to any location
- Fast and high-performance testing
- Low cost

In future work, we want to develop an application by using our model to perform the COVID-19 test. We also intend to adapt this solution to several other cases of diseases, pandemics, or epidemics.

## Figures and Tables

**Figure 1:** Proposed pipeline of our solution.

**Figure 2:** (a) Distribution of hematocrit variable. (b) Distribution of hemoglobin variable. (c) Distribution of platelets variable. (d) Distribution of mean platelet volume variable.

**Figure 3:** (a) Relation of the target and RSV variable. (b) Relation of the target and Influenza A variable. (c) Relation of the target and Influenza B variable. (d) Relation of the target and Parainfluenza 1 variable.

**Figure 4:** (a) Relation of the target and platelets variable. (b) Relation of the target and leukocytes variable. (c) Relation of the target and basophils variable. (d) Relation of the target and eosinophils variable.

**Figure 5:** Pipeline of the preprocessing.

**Figure 6:** Feature importance with ANOVA test.

**Figure 7:** Proposed pipeline of data modeling.

**Figure 8:** Proposed pipeline of optimization.

**Figure 9:** (a) Learning curves of random forest classifier. (b) Learning curves of bagging classifier. (c) Learning curves of AdaBoost classifier. (d) Learning curves of SVM. (e) Learning curves of KNeighbors classifier.

**Figure 10:** (a) Comparison between the five models in terms of accuracy. (b) Comparison between the five models in terms of sensitivity. (c) Comparison between the five models in terms of specificity.

**Figure 11:** Learning curves of the optimized best model according to the sample size.

**Figure 12:** (a) Comparison with the related works in terms of accuracy. (b) Comparison with the related works in terms of sensitivity. (c) Comparison with the related works in terms of specificity.

**Figure 13:** (a) Comparisons between models in terms of accuracy. (b) Comparisons between models in terms of sensitivity. (c) Comparisons between models in terms of specificity.

**Figure 14:** Difference between our model's performance and the one of [23].

**Table 1:** Summary of performance and description of related work.

Ref.	Dataset source	Dataset size	Total features	Model used	Accuracy	Sensitivity	Specificity
[23]	[24]	279	16	DT, ET, LR, RF, KNN, NB, SVM	82–86%	92–95%	—
[25]	[32]	599 (81)	108 (16)	Ensemble of 10 SVM models	—	70.25%	85.98%
[26]	[32]	598 (81)	108 (14)	RF, LR, GLMNET, ANN	81%–87%	43%–65%	81%–91%
[27]	[32]	253 (102)	108 (15)	NN, RF, GBT, LR, SVM	—	68%	85%
[28]	[32]	5644 (559)	108 (24)	XMLP, SVM, RT, RF, BN, NB	95.159%	96.8%	93.6%
[29]	[32]	5644 (279)	106 (97)	LR, NN, RF, SVM, XGB	—	80%	98%
[30]	—	5333 (160)	117 (35)	XGBoost, RF, DNN	—	81.9%	97.9%
[31]	[32]	5644	111	ET, RF, LR, XGBoost	99.88%	98.72%	99.99%
[33]	[32]	608	16	DTX, RF	88%	66%	91%
[34]	—	659	51	LASSO, Ridge, RF, XGBoost	—	92.5%	97.9%

**Table 2:** Values of the performance criteria.

	Accuracy	Sensitivity	Specificity
Random Forest	0.991	0.909	1
Bagging	0.988	0.909	0.997
AdaBoost	0.989	0.927	0.996
SVM	0.992	0.927	1
KNeighbors	0.990	0.909	0.999

**Table 3:** Confusion matrix of the optimized best model.

SVM	Predicted negative	Predicted positive
True negative	1018 (90.17%)	0 (0%)
True positive	8 (0.71%)	103 (9.12%)

## Data Availability

The data used to support this study are available in the following links: (1) https://www.kaggle.com/einsteindata4u/covid19; (2) https://zenodo.org/record/3886927#.YIluB5AzbMV.
